# The influence of bracket type on the external apical root resorption in class I extraction patients - a retrospective study

**DOI:** 10.1186/s12903-019-0743-3

**Published:** 2019-03-29

**Authors:** Fang Qin, Yu Zhou

**Affiliations:** 1 Department of Stomatology, Shaoxing People’s Hospital, Shaoxing, China; 2 Department of Orthodontic, School and Hospital of Stomatology, Wenzhou Medical University, Wenzhou, Zhejiang, China

**Keywords:** External apical root resorption, Passive self-ligating, Orthodontic, Conventional bracket

## Abstract

**Background:**

The relationship between orthodontic treatment-related factors and EARR has never been fully answered. The aim of this study was to investigate whether conventional and passive self-ligating brackets affect the amount and severity of external apical root resorption (EARR) in withdrawal patients.

**Methods:**

Ninety-eight patients were selected from department of orthodontic, hospital of stamotology, Wenzhou medical university. Patients received treatment with either a conventional edgewise appliance (*n* = 49, Mini, 3 M Unitek, USA) or a passive self-ligating bracket system (*n* = 49, Damon, Ormco, USA). EARR of the maxillary incisors was evaluated on panoramic radiographs at the before and end of orthodontic treatment, respectively. Intergroup comparisons of root resorption were performed with Mann-Whitney tests. The univariate and multivariate regression model was used to assess the appliance type, age, sex and duration of treatment on EARR.

**Results:**

There was no significant difference in the amount of EARR between the two groups was found. Age and gender were not association with EARR, however, EARR was positively correlated with treatment duration.

**Conclusions:**

The type of bracket did not influence the occurrence and severity of the external apical root resorption in class I extraction patients.

## Background

External apical root resorption (EARR) which defined as shortening or blunting of the root apex is considered as one of most serious adverse effect in orthodontic treatment [1]. The teeth of maxillary incisors are most prone to EARR [2].

However, the relationship between orthodontic and EARR has never been fully answered. Many factors, such as type of force application, treatment duration, force magnitudes and the distance of tooth movement, maybe contribute to the incidence and severity of EARR during orthodontic treatment [3–7].

In recently, many studies have come to a conclusion that mechanical forces play a key role in the occurrence of EARR during orthodontic treatment [8]. However, by now there were only few studies have assessed the effects of brackets type on EARR [9–12]. Self-ligating brackets have been gaining popularity in recent years which was first introduced in the early 1930s [11]. These brackets claimed advantages of shorter treatment time, less friction and a higher rate of teeth movement. Because of so many advantages, a hypothesis has been raised as to their effect on EARR. But, the occurrence of EARR between conventional and passive self-ligating brackets has not yet been fully investigated. In the orthodontic literatures, there are few studies have explored the influence of self-ligating brackets on EARR [9–12]. Previous studies found that no significant difference regarding the occurrence of EARR between conventional and passive self-ligating brackets. However most of these studies shortage were a small amount of patients or with different treatment plan [9–12]. As I known, this is the first study which only included extraction patient to assess the amount and severity of external apical root resorption. Thus, the purpose of this study was to investigate the incidence of EARR on maxillary incisors in extraction patients treated with conventional brackets and passive self-ligating brackets. We furthermore analyze the influence of age, gender and treatment time on the occurrence of EARR.

## Materials and methods

### Patients

According to the previous study, in order to detect a significant change in root resorption we need a sample size of 42 subjects, with an 80% probability power at the 5% level of significance.

In this retrospective study, 98 participants were selected from 489 patients who completed the orthodontic treatment in the Department of orthodontic, hospital of stomatology, Wenzhou Medical University. They were divided into two groups: passive self-ligating brackets group (Damon 3, OMRCO, USA) and conventional brackets group (3 M Unitek, California, USA). The inclusion and exclusion criteria see Table 1. The demographics of these subjects are listed in Table 2.

**Table 1:** Inclusion and exclusion criteria in two groups

Inclusion criteria	
1. completed orthodontic treatment with SL or CL brackets, and not receive orthodontic treatment before 2. panoramic radiograph before and after treatment 3. completed root growth of the maxillary incisors before treatment 4. no evidence of EARR of the maxillary incisors on the pretreatment panoramic radiograph 5. no severely dilacerated incisor roots 6. class I molar relationship before treatment and extract four first premolar 7. No root canal teeth, prosthesis	
Exclusion criteria	
1. impacted teeth 2. trauma before and during orthodontic treatment 3. caries or periodontal disease 4. other systemic diseases, such as lip\palatal cleft

**Table 2:** Demographic and clinical characteristics of the patients in two groups

Characteristics	Conventional (mean and SD)		Self-ligating (mean and SD)		*P* value
Age	15.21	4.43	15.15	4.52	NS
Sex					
Female	23		24		
Male	26		25		NS
Treatment duration (mo)	22.10	5.15	20.25	5.11	NS

### Treatment procedure

The archwire sequence was 0.012-in, 0.016-in and 0.019 × 0.025-in copper- nickel-titanium (Ormco) and finished with 0.019 × 0.025-in stainless steel in conventional group. The archwire sequence for the self-ligating group included 0.014-in, a 0.014 × 0.025-in copper-nickel-titanium Damon (Ormco) and finished with 0.019 × 0.025-in stainless steel. All the patients were treated by the same clinician who has received training in both appliance systems.

The panoramic radiographs were taken before and after treatment with the same radiographic machine (SIEMENS, SIDEXIS XG, Germany) and by the same operator.

### X-ray measurement and patient informed consent

Correction Factor (CF) = C1/C2.

C1 = Crown length on pretreatment radiograph

C2 = Crown length on post-treatment radiograph

The measurement of EARR as following.

R1 = Root length before treatment

R2 = Root length after treatment

The relative root resorption (rRR) which seen as the percentage shortening per tooth was used to represent the EARR, see Fig. 1.

**Fig. 1:** X-ray measurement of root resorption. Reference points:1 root apex,2 distal dento-enamel junction,3 mesial dento-enamel junction,4 incisal edge. Dento-enamel conjunction (DEC) represents the conjunction between mesial and distal. Crown length(C) and root length(R) were measured perpendicular to DEC as the longest distance to the root apex and the incisal edge. This figure first describe by Jacobs et al. Head & face medicine 2014,10:2

Quantitative measurements of the crown and root length of the maxillary central and lateral incisors were taken. The crown length registrations was used to assess the image distortion between the before and after treatment radiographs. Linge and many other study had described this measurement method in previous studies [13, 14] (Fig. 2).

**Fig. 2:** External apical root resorption (EARR) stages according to Malmgren et al. 1 irregular root contour, 2 EARR< 2 mm of root length, 3 EARR > 2 mm to 1/3 of root length, 4 EARR> 1 /3 of root length. This figure was first described by Jacobs et al. Head & face medicine 2014,10:2

The calibrated panoramic radiographs were used to measure incisor root lengths before and after treatment. All patients were informed about the purpose of this research and given their informed consent.

### Statistical assessment

The pair-T or chi-square test were conducted to examine the difference between two groups. The multiple regression models were used to investigate the factors of EARR, such as gender, age, and treatment duration. The significance level was set at 0.05. All statistical analyses were performed using SPSS 20.0 (SPSS Inc., Chicago IL, USA).

### Error determination

According to Dahlberg’s formula [15], 20 panoramic radiographs were randomly retraced and were re-measured 2 months after the first assessment to determine systematic error. The error results fell within a very good range of (0.12 mm).

## Results

Table 2 shows the baseline information of 2 appliance groups. There was no significance difference in baseline information between the two appliance groups.

In Table 3, all teeth occurred root resorption and reached a statistically level after treatment in group I. In Table 4, we can see that the same situation in Group II. However, in Table 5, there was no statistically significant difference was found between the two groups in the degree of root resorption.

**Table 3:** The degree of root resorption (mm) between T1 and T2 for the patients in self-ligating brackets group

Measurements, mm	T1		T2		T2–T1	P
	Mean	SD	Mean	SD		
Maxillary right central incisor	25.23	1.58	24.91	1.28	−0.32	0.001
Maxillary right lateral incisor	24.35	1.26	24.08	1.22	−0.27	0.001
Maxillary left central incisor	25.25	1.54	24.92	1.32	−0.33	0.004
Maxillary left lateral incisor	24.27	1.25	23.99	1.35	−0.28	0.001

**Table 4:** The degree of root resorption (mm) between T1 and T2 for the patients in conventional preadjusted brackets group

Measurements, mm	T1		T2			
	Mean	SD	Mean	SD	T2–T1	P
Maxillary right central incisor	25.26	1.26	24.86	1.18	−0.40	0.002
Maxillary right lateral incisor	24.52	1.32	24.17	1.29	−0.30	0.007
Maxillary left central incisor	25.22	1.52	24.83	1.24	−0.39	0.001
Maxillary left lateral incisor	24.54	1.26	24.23	1.35	−0.31	0.005

**Table 5:** The Difference in Root resorption between Self-ligating brackets and conventional brackets group

Measurements, mm	Self-ligating Brackets Group		Conventional Brackets Group		P
	Mean	SD	Mean	SD	
Maxillary right central incisor	−0.32	0.24	−0.40	0.28	NS
Maxillary right lateral incisor	−0.27	0.28	−0.30	0.25	NS
Maxillary left central incisor	−0.33	0.27	−0.39	0.31	NS
Maxillary left lateral incisor	−0.28	0.25	−0.31	0.26	NS

In Table 6, we found that self-ligating bracket group had 49% and conventional bracket group had 35% of the teeth classified with scores of 0 and 1. When refer to the score of 2 to 4, group 1 had 51% and group 2 had 65%.

**Table 6:** Distribution of teeth with apical root resorption

Score	Self-ligating Brackets Group		Conventional Brackets Group		P
	n	%	n	%	
0	4	8	5	10	
1	20	41	12	25	
2	18	37	20	41	
3	4	8	7	14	
4	3	6	5	10	NS

Table 7 showed that EARR increased when treatment duration increased by using univariate analysis. Multivariate regression showed that treatment duration was significant risk factors of EARR. Extension of treatment time by 1 month will lead to root absorption of 0.05 mm. Compared to self-ligating brackets, conventional appliances induced more EARR with an average of 0.35 mm when take treatment duration effects into accounting (Table 7).

**Table 7:** Predictor factors for root resorption (mm) as dependent variable by using univariate and multivariate model

Predictor variables	Category	Univariate model			Multivariate model		
		b	SE	*P* value	b	SE	*P* value
Appliance	Conventional	baseline			baseline		
	Self-ligating	0.42	0.22	NS	0.35	0.16	0.04
Treatment duration	1 month	0.05	0.01	0.03	0.05	0.04	0.02
Sex	Female	baseline					
	Male	0.32	0.45	NS			
Age	1 year	0.24	0.18	NS			

## Discussion

In this study, we are aimed to investigate the amount of EARR and the occurrence of EARR on maxillary incisors in extraction patients between SL and Non-SL brackets. We found that there is no difference in the amount of EARR between conventional and passive self-ligating brackets group. To our best knowledge, this is the first study which only included extraction patients to assess the amount of EARR between conventional and passive self-ligating brackets. In the previous studies [9–11], they were included patients with or without extraction when assess the occurrence of EARR. We all know that patients with tooth extraction are more prone to root resorption than those without tooth extraction [16–18]. It is not wise to combine the extraction and non-extraction patients for analysis in one study.

Compare to the previous studies, in this study, all patients were treated by one orthodontist with the similar sequence of changing archwires. This guarantees a good comparability between the two groups. Furthermore, we recruited more patients than previous studies, which may display a higher value of significance [9–11].

This study only included maxillary incisors because maxillary incisors were most susceptible to root resorption during orthodontic treatment. The results of this study found that an average of 0.3 mm and 0.35 mm root resorption in conventional bracket and self-ligating group groups, respectively. Other studies found the average of root resorption were range from 0.53 mm to 0.76 mm in fixed appliance [19–22]. The reason may be the different measure method and the included different patients.

Compared with conventional brackets, it has been hypothesized that fast tooth movement in self-ligating brackets will result in more EARR during the orthodontic treatment [23, 24]. However, in this study, we found that there was no statistically significant difference between conventional and self-ligating brackets group in EARR. Multivariate regression also showed that appliance type was not significant risk factors of EARR. Others studies also confirmed the same results that self-ligating brackets did not lead to the higher rate of EARR [9–12].

There was no significance difference between two groups in relative severe root resorption, but the number of severe root resorption was less in self-ligating brackets than conventional brackets group. The explanation may be due to the continuous light force provided by the self-ligating brackets. Light forces have long been recommended to reduce adverse tissue reactions, such as root resorption [25].

In this study, we are interested to find that treatment during is a predictor factor of EARR when receive the orthodontic treatment. We are even further come to a conclusion that extension of treatment time by 1 month will lead to root absorption of 0.05 mm. The reason may be extended tooth movement will result in persistent bone turnover which may cause more root resorption [26]. Others also found the treatment duration had a positive association with the amount of EARR [27, 28].

Some deficiencies still need to draw our attention. First, the panoramic radiographs is not precise than periapical radiographs or CBCT for measuring EARR [29]. However, taking into account that the higher radiation dose of the periapical radiographs or CBCT, and many studies have confirmed that it is possible to use a panoramic film to initially determine the amount of root absorption [30–32]. Second, although we strictly matched the treatment group and the control group when selecting cases, it may be difficult to avoid the influence of confounding factors on the results. It is better to adopt randomize design to compare the EARR between the two type brackets in the future. At last, we still need to include more different ethnic patients to verify whether the two brackets influence the root resorption.

## Conclusions

There was no statistically significant difference in the occurrence of EARR and the amount of EARR between conventional and passive self-ligating brackets in class I extraction patients.

## Abbreviations

EARR: External apical root resorption
SL: Self-ligating bracket
